The article "Exoskeleton Follow-Up Control Based on Parameter Optimization of Predictive Algorithm" was published in 2021. Journal: Appl Bionics Biomech.

# Exoskeleton Follow-Up Control Based on Parameter Optimization of Predictive Algorithm

**DOI:** 10.1155/2021/8850348

**Published:** 2021-01-21

**Authors:** Shijia Zha, Tianyi Li, Lidan Cheng, Jihua Gu, Wei Wei, Xichuan Lin, Shaofei Gu

**Affiliations:** ^1^College of Optoelectronics Science and Engineering, Soochow University, Suzhou Jiangsu Province, 215000, China; ^2^Micro-Nano Automation Institute, Jiangsu Industrial Technology Research Institute, Suzhou, Jiangsu Province 215131, China; ^3^Shanghai Huangpu District Fire Rescue Detachment, Shanghai 200001, China

## Abstract

The prediction of sensor data can help the exoskeleton control system to get the human motion intention and target position in advance, so as to reduce the human-machine interaction force. In this paper, an improved method for the prediction algorithm of exoskeleton sensor data is proposed. Through an algorithm simulation test and two-link simulation experiment, the algorithm improves the prediction accuracy by 14.23 ± 0.5%, and the sensor data is smooth. Input the predicted signal into the two-link model, and use the calculated torque method to verify the prediction accuracy data and smoothness. The simulation results showed that the algorithm can predict the joint angle of the human body and can be used for the follow-up control of the swinging legs of the exoskeleton.

## 1. Introduction

The exoskeleton is a wearable device that combines human intelligence and mechanical power, widely appearing in the fields of assistance, rehabilitation training, and disability assistance. In recent years, with the continuous development of drive technology and sensor technology, more and more exoskeletons have appeared in the market [1]. Exoskeletons are often designed to perform specific functions such as walking, weight-bearing, lumbar support, and spinal support. In order to assist the specific movements of the human body, a very critical point for the exoskeleton is to realize the recognition of the human motion intention.

### 1.1. Introduction to Exoskeleton Classification

There are many ways to classify active exoskeletons. One classification way is based on the methods of the exoskeleton acquiring the intention of human motion, which can be roughly divided into four categories: The first is preprogrammed. The gait of the exoskeleton system is designed, so the wearer can only intervene in limited ways with devices such as buttons or HMI (Human Machine Interface). However, only relying on some external devices to obtain the motion intention of the human body limits the use scope of the exoskeleton, which makes this kind of exoskeleton often appear in the rehabilitation and correction equipment with fixed gait [2]. The second is the use of EEG (electroencephalogram) signals to identify the intention of human movement. Such systems are susceptible to interference from the external environment and are not suitable for the wearer to perform multibrain tasks [3]. The third method uses the surface EMG (electromyography) signals of the human body to capture the movement intention of the human body. Obtaining surface EMG signals is usually done by attaching electrodes on the skin of the human body, which is also vulnerable to the environment. Sweat on the surface of the skin often affects the accuracy of the signals [4], and long-term wear is easy to cause the surface electrode to fall off; some teams have developed exoskeletons (e.g., HAL) that recognize the body's intentions based on electromyographic signals. The fourth way is to collect human body motion mechanics information to identify human body motion intentions. Such systems have installed a large number of kinematics and dynamics sensing devices on the exoskeleton and human body to obtain the interaction information of the human body and the motion intention of the human body. Many lower limb exoskeletons, such as WEAR [5], MEBOTX-EXO [6], and HUALEX [7], use kinematic information to capture the human body's intention and kinetic information to control the motion of the exoskeleton. This type of exoskeleton has the characteristics of easy to put on and take off, and the system sensor signal is stable, which makes it become the main research direction of exoskeleton. However, the kinematic sensor requires the human body to drive the exoskeleton movement, inevitably causing the delay of motion intention perception and control.

Since the exoskeleton involved in this paper is the fourth method to obtain the human movement intention and the sensor data is collected by the sensor network, it takes some time until the control signal is generated. The actuators (typically motors or hydraulic) cause time delay, too [8]. Meanwhile, the motion signal of the human body is behind the motion intention of the human body. Therefore, it is necessary to solve the time delay in the fourth exoskeleton system.

### 1.2. Introduction to Prediction Algorithm

In the exoskeleton control strategies, only relying on the sensor data detected by the sensors of the system and giving the exoskeleton drive structure motion instruction will cause the exoskeleton and the human body a position deviation. The position deviation is the main source of human-machine interaction. An appropriate prediction algorithm needs to be added to help the control strategies judge the wearer's motion intention and the possible motion position at the next moment according to the current and historical motion sensing data, so as to give the system appropriate control commands. Due to the significant difference in the delay between the exoskeleton and the wearer due to different wearing methods and the tightness of the binding, some prediction methods can only predict the one step size, such as Kalman prediction [9], need to continuously iterate the Kalman gain coefficient according to the measured value, and cannot deal with the longer step size prediction. Similar problems also exist in the prediction methods based on the ARMA model, such as LMS linear prediction [10] and RLS linear prediction [11, 12]. When the prediction step size becomes longer, the accuracy of the prediction will decrease significantly [13]. Moreover, LMS linear prediction and RLS linear prediction require more historical data and a large amount of computation, and the prediction curve is not smooth, which makes it difficult to implement such prediction algorithm in an embedded system.

Yang [13] et al. compared the performance of LMS and Takens prediction algorithms in the prediction of human gait data. The results showed that Takens is more stable, accurate, and suitable than LMS, but it did not solve the zero dead time problem of the prediction algorithm. So, Duan et al. [14] use the combination of the Takens prediction algorithm and Newton-based-method to solve the problem of the zero dead time of the prediction algorithm but did not make progress in solving the parameter tuning process.

In this work, we have made improvements to the prediction algorithm for exoskeleton, so that the parameters of the prediction algorithm can be optimally determined. Applying it to exoskeleton gait prediction can accurately predict the joint angle of the exoskeleton, making joints motor reach the aim position in advance.

The reminder of this paper is organized as follows:

In Section 2.1, we introduce the IMU-based pose capture system. In Section 2.2, we briefly introduce the Takens prediction algorithm. In Section 2.3, we introduce the process of the PSO-Takens algorithm.  Section 2.4 is mainly about the simulation of the control of the prediction algorithm in the two-link model.

In Section 3, the experimental results are analyzed. We mainly discussed the performance of the improved prediction algorithm and the original prediction algorithm in exoskeleton gait data prediction.

In Section 4, we conclude the paper.

## 2. Materials and Methods

### 2.1. Motion Capture System

The process of human lower limb movement has the characteristics of high autonomy, complex information, diverse movements, and multiple degrees of freedom. Biomechanical simulation and experimental studies have shown that the motion consumption power in the sagittal plane of the human body is the largest relative to the frontal plane and horizontal plane [15], so the three-dimensional walking motion of human hip joint often can be simplified to a single plane motion in the sagittal plane. The corresponding position sensor used in the exoskeleton is usually placed in a position parallel to the sagittal plane of the human body, which describes the motion angle of the sagittal plane of the lower limb joints of the human body. With the development of inertial measurement units, more and more IMUs (inertial measurement units) were used as examples of kinematic sensors, beginning to appear in the motion capture system. Compared with the method of collecting joint angles using an absolute encoder, IMU has an advantage of flexible installation and cheap price, and its measurement accuracy can reach 0.1°, which can meet the needs of the human motion capture system.

In order to collect human gait information and verify the accuracy of the prediction algorithm, we designed a flexible motion capture system for human sagittal plane motion based on IMUs. The system will automatically capture the sagittal plane motion data of the human body at 50 Hz sampling frequency and transmit the motion data through CAN (Controller Area Network) (Figure 1(a)) to the data collection and processing module. As shown in Figure 1(b), the system mainly collected the pitch angle data of the back, thigh, shank, and the pressure sensor data of the heel. The system also includes power module, data collection and processing module, and data transmission module.  Figure 1(c) shows the actual mechanical structure of the exoskeleton system, a hinged structure is adopted between the thigh and shank, and this structure can support the exoskeleton system and reduce the load on the body while standing upright, but it also leads to the inability to directly measure the motion angle of the human knee joint through the angle sensor. Therefore, IMUs were placed on the thighs, shanks, and back to calculate the angle of the human joints.

The formula for calculating the angle of the hip and knee joints is as follows:

(1) $$\begin{array}{c} \theta_{\text{hip}}=\frac{\pi }{2}-\theta_{h},\\ \theta_{\text{knee}}=\pi -\theta_{h}-\theta_{l}. \end{array}$$

 *θ*_*h*_, *θ*_*l*_ represents the pitch angle of thigh and shank, respectively; due to the mirror relationship between the left and right legs, the calculated angle values are opposite, and there is a phase difference between the hip joints and knee joints.

### 2.2. Takens Prediction Algorithm

The continuous walking of the human body is periodic and nonlinear. The left and right leg sensor data are only different in phases and directions. Therefore, the algorithms used in the prediction of the joint angle are the same; the prediction algorithms discussed in this section are nonlinear time series Takens prediction algorithm of the lower limb hip and knee joint data.

The Takens algorithm for nonlinear time series forecasting is based on the Takens embedding theorem, which is also called the weighted zero-order local prediction method. This method is closely related to Takens' reconstruction theorem. It is essentially a nonlinear time series analysis method, which requires historical data of the system to obtain the best performance. The main idea is to find several historical data vectors that are the most similar to the current reconstruction delay vector by traversing the sensor data for a period of time, and the historical data vector is normalized and weighted according to the similarity with the current sampling data. The prediction data at a specific time is determined through function fitting or search. The predicted data of each vector are multiplied by their respective weights to obtain the final predicted value at the determined moment. The algorithm implementation steps are as follows:

(1) According to the Takens embedding theorem, for a given time series *y*(*t*), select the appropriate sampling interval ∆*t* and embedding dimension *n*, and collect and store *n* data; the adjacent data differ in time ∆*t*; constitute the reconstruction delay vector *D*(*t*). The time series *y*(*t*) can be any type of sensor data in the motion capture system, such as angle, angular velocity, or heel pressure data. The contents of *D*(*t*) is
  (2) $$\begin{array}{c} D\left(t\right)=\left[y\left(t\right),y\left(t-\Delta t\right),y\left(t-2\Delta t\right),y\left(t-3\Delta t\right)\cdots y\left(t-\left(n-1\right)\Delta t\right)\right] \end{array}$$
(2) Calculate the similarity between the current reconstruction delay vector *D*(*t*) obtained by sampling at the current time and the historical reconstruction delay vector *D*_*i*_(*t*) obtained from all previous observations; the methods for calculating similarity in reconstruction delay vectors are usually Euclidean distance, Pearson's correlation coefficient, Manhattan distance, and hash distance. The Euclidean distance has the following expression in this algorithm:
  (3) $$\begin{array}{c} \delta \left(i\right)=\sqrt{\overset{n}{\underset{k=1}{\sum }}{\left(y\left(t-\left(k-1\right)\Delta t\right)-y_{i}\left(t-\left(k-1\right)\Delta t\right)\right)}^{2}}\;\left(1\leq i\leq N\right). \end{array}$$

In formula (3), the value of *i* represents the position of the currently traversed vector, N is the reconstruction delay vector length. The smaller the Euclidean distance is, the more similar the two reconstruction delay vectors are, and the more accurate when the historical reconstruction delay vector is used to predict the data of the subsequent period of time. While Pearson's correlation coefficient or Manhattan distance is used as a similarity calculation, the expression becomes

(4) $$\begin{array}{c} \delta \left(i\right)=\frac{\sum_{k=1}^{n}\left(y\left(t-\left(k-1\right)\Delta t-\bar{y}\right)\left(y_{i}\left(t-\left(k-1\right)∆t-\bar{y_{i}}\right)\right)\right)}{\sqrt{\sum_{k=1}^{n}{\left(y\left(t-\left(k-1\right.\right)\Delta t-\bar{y}\right)}^{2}}\sqrt{\sum_{k=1}^{n}{\left(y_{i}\left(t-\left(k-1\right)∆t-\bar{y_{i}}\right)\right)}^{2}}}\;\left(1\leq i\leq N\right),\\ \delta \left(i\right)=\overset{n}{\underset{k=1}{\sum }}\left|y\left(t-\left(k-1\right)\Delta t\right)-y_{i}\left(t-\left(k-1\right)\Delta t\right)\right|\;\left(1\leq i\leq N\right). \end{array}$$

In formula (4), $\bar{y}$ is the average value of the reconstructed delay vector, Pearson's correlation coefficient and Manhattan distance can also be used as a similarity calculation function, and the difference is only the amount of calculation. Among the three calculation methods, Manhattan has the smallest amount of calculation and Pearson's correlation coefficient is the largest

(3) From the observed historical reconstruction delay vector *D*_*i*_(*t*), the best matching M sets of reconstruction delay vectors {*D*_1_(*t*), ⋯, *D*_*M*_(*t*)} are selected according to the similarity with the reconstruction delay vector *D*(*t*) at the current moment. The corresponding Euclidean distances are {*δ*(1), ⋯, *δ*(*M*)}. The predicted value {*y*_1_(*t* + *b*∆*t*), ⋯, *y*_*M*_(*t* + *b*∆*t*)} of each group of reconstruction delay vectors is determined by searching, *T* = *b*∆*t* is the predicted duration. The weighting factor formula of each best matching amount in the final prediction amount calculation formula is as follows:
  (5) $$\begin{array}{c} w_{i}=\frac{1}{\sum_{j=1}^{M}\delta_{i}}\frac{1}{\delta_{i}}\;\left(1\leq j\leq M\right) \end{array}$$
(4) According to the predicted values and weight factors of each historical reconstruction delay vector group, the estimated predicted values at time *b*∆*t* after the current moment *y*(*t*) are calculated as follows:
  (6) $$\begin{array}{c} \hat{y}\left(t+b\Delta t\right)=\overset{M}{\underset{i=1}{\sum }}w_{i}y_{i}\left(t+b\Delta t\right) \end{array}$$

The flow chart of the algorithm is shown in Figure 2.

The Takens algorithm is to make predictions on the sensor data for a period of time by searching historical sensor data, which means that the prediction algorithm is to find the most similar data out of the current motion situation from the historical vectors. The sensor data of the human walking motion detected on the sagittal plane has obvious periodicity, so the Takens algorithm has a well performance in predicting such signals. Among multiple optimal reconstruction delay vectors, the algorithm can dynamically adjust the weight factor through the Euclidean distance, which can adjust the proportion of the optimal reconstruction delay vector in the final prediction data.

### 2.3. PSO-Takens Prediction Algorithm Design

Although the Takens algorithm cannot predict that all motion sensor data are completely correct, some papers also give an optimization method based on this algorithm [14], which makes the Takens algorithm used in embedded systems become possible. Whitney's topological embedding theorem shows that the phase space of the original system can be reconstructed by any value of the delay time of the single variable time series in the case of noiseless and infinitely long time series. In fact, the measured time series is of limited length and is inevitably polluted by noise. Therefore, arbitrary delay time cannot reconstruct the phase space of the system; the key to reconstruct the phase space using the measured time series is how to select these reconstruction parameters. However, the Takens embedding theorem does not indicate how to select these parameters. This problem has become an important issue in nonlinear time series analysis.

Duan et al. have found that inappropriate historical vector dimension and embedding dimension will cause irrelevant data to enter the reconstruction delay vector, resulting in lower prediction accuracy [14]. While inappropriate prediction duration and optimal matching number will cause data jitter and affect the smoothness of the predicted data. Fortunately, the predicted duration, which is also called delay time, is a constant we want to compensate. It is mainly caused by inertial sensors and inherent defects of the system, and the duration can be measured by wearing exoskeletons. The delay time is expressed as the angle difference between the human body and the exoskeleton.

In order to evaluate the algorithm performance and adjust the parameters of the algorithm, the following two formulas were introduced which are aimed at judging the pros and cons of the prediction effect:

#### 2.3.1. Prediction Accuracy Rate (PR)

(7) $$\begin{array}{c} e_{k}\left(t\right)=y\left(t\right)-\hat{y}\left(t\;|\;t-b\Delta t\right),\\ \text{RMS}\left(e_{k}\right)=\sqrt{\frac{1}{n}\overset{n}{\underset{t=2}{\sum }}e_{k}{\left(t\right)}^{2}}. \end{array}$$

*e*_*k*_(*t*) records the error between the predicted value and the actual value at each sampling point, and RMS(*e*_*k*_) (Root Mean Square error) characterizes the degree of deviation of the overall predicted value from the actual value. The greater the RMS(*e*_*k*_) is, the greater the deviation of the predicted data from sensor data and the worse the predicted performance. By normalizing the RMS(*e*_*k*_), the prediction accuracy rate (PR) is defined as

(8) $$\begin{array}{c} \text{PR}\left(y\left(t\right),e_{k}\left(t\right)\right)=1-\frac{\text{RMS}\left(e_{k}\left(t\right)\right)}{\text{RMS}\left(y\left(t\right)\right)}\times 100\%. \end{array}$$

#### 2.3.2. Smooth Factor (SF)

(9) $$\begin{array}{c} \text{SF}\left(\hat{y}\left(t\right)\right)=\frac{1}{t_{\text{end}}\left(\max\left(\hat{y}\left(t\right)\right)-\min\left(\hat{y}\left(t\right)\right)\right)}\int_{0}^{t_{\text{end}}}\left|f\left(t\right)-\hat{y}\left(t\right)\right|. \end{array}$$

In formula (9), *t*_end_ is the duration of the algorithm, and a 5 Hz low-pass filter is used to filter *y*(*t*) to obtain *f*(*t*). The parameter smooth factor (SF) indicates whether the data is smooth or not. In the course of human gait walking, the predicted sensor data is smooth and stable to match the actual walking data. Therefore, the smaller the SF is, the closer the predicted sensor data is to the sensor data measured by the actual gait walking. Since the data actually collected in the algorithm is discrete, when calculating the SF, formula (12) is usually discretized to the following formula:

(10) $$\begin{array}{c} \text{SF}\left(\hat{y}\left(t\right)\right)=\frac{1}{N\left(\max\left(\hat{y}\left(t\right)\right)-\min\left(\hat{y}\left(t\right)\right)\right)}\overset{N}{\underset{i=0}{\sum }}\left|f\left(i\right)-\hat{y}\left(i\right)\right|. \end{array}$$

The parameters affecting the prediction effect of the Takens algorithm are as follows: (i) the predicted duration (*T*), (ii) historical reconstruction delay vector length (*P*), (iii) optimal matching reconstruction vector number (*M*), and (iv) embedding dimension (*N*).

We introduced PSO (Particle Swarm Optimization) on the basis of Takens prediction algorithms, which is a swarm intelligence optimization algorithm in addition to an ant colony algorithm and a genetic algorithm in the field of computer intelligence. It originated from the study of bird predation behavior, and the basic idea is to solve and cooperate with individuals in the group to achieve the search for the optimal solution in a complex space [16]. Compared with other intelligent adjustment algorithms [17–18], such as derivative-based or derivative-based (or gradient-based) (e.g., backpropagation (BP), Levenberg-Marquardt (LM), Kalman filter, least square methods, and sliding-mode learning algorithm), hybrid learning methods, it belongs to the derivative-free method and does not need to update complex parameter equations, making it more suitable for nonlinear output situations. Meanwhile, it has the advantages of strong global search ability and easy implementation and has strong convergence and robustness in the process of solving. In the PSO algorithm, each particle represents a potential solution, and the velocity of the particle represents the direction and distance of each potential solution, which can be used to seek the optimal value in the multidimensional space.

The PSO-Takens algorithm flow chart is shown in Figure 3.

**Step 1 .**

Initialize a swarm of particles (population size *m*), including the random position and velocity, and limit the upper and lower limits of the particle's velocity and position. The optimized parameters in the Takens algorithm are as follows: historical vector dimension *P*, optimal matching number *M*, and embedding dimension *N*; therefore, the population of particles is {*x*1, *x*2, *x*3 ⋯ *Xm*}, and the position of the *i*-th particle is {*XP*_*i*_, *XM*_*i*_, *XN*_*i*_}, The velocity of the *i*-th particle is {*VP*_*i*_, *VN*_*i*_, *VM*_*i*_}.

**Step 2 .**

Use the evaluation function to calculate the fitness of each particle.

**Step 3 .**

For each particle, comparing its fitness with the optimal value *p*best, it has passed through. If the current value is better than *p*best, the *p*best will be set to the current value, and the position of *p*best is set as the current position in the *n*-dimensional space.

**Step 4 .**

For each particle, comparing its fitness value with the best position *g*best, all particles passed through. If the current value is better, the current position will be regarded as the best position *g*best.

**Step 5 .**

After updating the local and global optimal values of the current iteration, the particle adjusts its velocity and position through the following formulas.

(11) $$\begin{array}{c} V_{i+1}=V_{i}+c_{1}\times r\text{and}\left(\right)\times \left(p\text{bes}{\text{t}}_{i}-x_{i}\right)+c_{2}\times r\text{and}\left(\right)\times \left(g\text{bes}{\text{t}}_{i}-x_{i}\right),\\ x_{i+1}=x_{i}+V_{i+1}. \end{array}$$

When the inertia factor is added, the velocity expression becomes

(12) $$\begin{array}{c} V_{i+1}=\omega V_{i}+c_{1}\times r\text{and}\left(\right)\times \left(p\text{bes}{\text{t}}_{i}-x_{i}\right)+c_{2}\times r\text{and}\left(\right)\times \left(g\text{bes}{\text{t}}_{i}-x_{i}\right). \end{array}$$

**Step 6 .**

If the condition to terminate the iteration is not reached, go to Step2, until the iteration termination condition is met.

According to the specific issue, the iteration termination condition is generally to reach the maximum iteration number *Gk* or the optimal value of the evaluation function to meet the established threshold. The condition for the algorithm to stop iteration is as follows: the number of iterations over 50, or the fitness calculated by the evaluation function over 100. The fitness (*Y*_ef_) evaluation function expression is follows:

(13) $$\begin{array}{c} Y_{\text{ef}}=w_{1}\times \frac{1}{\text{SF}}+w_{2}\times \text{PR}. \end{array}$$

In formula (15), *w*_1_ and *w*_2_ are constants (0.5), which means that we believe that the accuracy of data is as important as the smooth factor in the human lower limb prediction algorithm. The goal of the PSO-Takens prediction algorithm is to adjust the complex parameter tuning problem of the Takens algorithm in gait prediction, so as to achieve the optimal prediction effect.

### 2.4. Follow-Up Control Design

#### 2.4.1. Dynamic Model of Swing Leg

The movement of the lower limbs of the human body can be regarded as a combination of swing phase and support phase. Usually, the swing phase accounts for 60% of the gait cycle and the support phase accounts for 40% [19]. For the swinging phase, the swinging legs of the human body can be regarded as an inverted two-link with uniform mass distribution. During the support phase, the leg and the upper body of the human body can be regarded as three links fixed at the bottom. This division method can simplify the complexity of torque calculation in inverse dynamics, making it easy to implement on embedded systems.

The lower limb-assisted exoskeleton single leg model is shown in Figure 4. *L*_0_ and *L*_1_ are the length of thigh and shank, and the ankle joint is omitted.

Assuming that the mass distribution of the exoskeleton lower limb members is uniform, the centroid coordinates *G*_*i*_(*x*_*i*_, *z*_*i*_) of the exoskeleton thigh and shank are as follows:

(14) $$\begin{array}{c} \left\{\begin{array}{c} x_{0}=a_{0}\sin q_{0,}\\ z_{0}=-a_{0}\cos q_{0,} \end{array}\right. \end{array}$$

(15) $$\begin{array}{c} \left\{\begin{array}{c} x_{1}=L_{0}\sin q_{0}+a_{1}\sin q_{1,}\\ z_{1}=-\left(L_{0}\cos q_{0}+a_{1}\cos q_{1}\right). \end{array}\right. \end{array}$$

The kinetic energy of the two connecting rods of lower limb swing is the sum of the rotational kinetic energy and kinetic energy of the connecting rod, which can be expressed as follows:

(16) $$\begin{array}{c} E=\frac{1}{2}\left(\overset{1}{\underset{i=0}{\sum }}I_{i}{\ddot{q}}_{i}+m_{i}\left({{\dot{z}}_{i}}^{2}+{{\dot{x}}_{i}}^{2}\right)\right). \end{array}$$

In formula (16), *I*_*i*_ is the moment of inertia when the exoskeleton is the *i*-th lower extremity connecting rod rotating around the sagittal plane of the joint. The expression is *I*_*i*_ = (1/3)*m*_*i*_*L*_*i*_^2^, and ${\ddot{q}}_{i}$ is the angular acceleration of the joint. ${\dot{z}}_{i}\text{ and }{\dot{x}}_{i}$ are the velocities of the linkage in the *x* and *z* directions, and the total potential energy of the lower limb linkage is as follows:

(17) $$\begin{array}{c} P=\overset{1}{\underset{i=0}{\sum }}m_{i}gz_{i}. \end{array}$$

By defining the Lagrangian function *L* = *E* − *P* and the Lagrangian formula, the expression of the joint torque in the two-link can be expressed as

(18) $$\begin{array}{c} H\left(q\right){\ddot{q}}_{i}+C\left(q,\dot{q}\right)\dot{q}+G\left(q\right)=\tau_{i}. \end{array}$$

In formula (18), *τ*_*i*_ is the joint torque between the links, *H*(*q*) is the inertia matrix, $C\left(q,\dot{q}\right)$ is the friction matrix, and *G*(*q*) is the gravity vector. The expressions of the matrix *H*(*q*), $C\left(q,\dot{q}\right)$, and the gravity vector *G*(*q*) are as follows:

(19) $$\begin{array}{c} H\left(q\right)=\left[\begin{array}{cc} \frac{7}{12}m_{0}l_{0}^{2}+m_{1}l_{1}^{2} & m_{1}l_{0}l_{1}\cos\left(q_{0}+q_{1}\right)\\ 0 & \frac{7}{12}m_{1}l_{1}^{2} \end{array}\right],\\ C\left(q,\dot{q}\right)=\left[\begin{array}{cc} 0 & -m_{1}l_{0}l_{1}\sin\left(q_{0}+q_{1}\right)\\ -m_{1}l_{0}l_{1}\sin\left(q_{0}+q_{1}\right) & 0 \end{array}\right],\\ G\left(q\right)=\left[\begin{array}{c} \frac{1}{2}m_{0}gl_{0}\sin q_{0}+m_{1}gl_{0}\sin q_{0}\\ \frac{1}{2}m_{1}gl_{1}\sin q_{1} \end{array}\right]. \end{array}$$

#### 2.4.2. Follow-Up Control Strategy

After obtaining the inverse dynamics model of the joint, we use the prediction angle obtained by the prediction algorithm to do Simulink simulation of the two-link model in MATLAB. The follow-up control strategy block diagram is shown in Figure 5.

The input of the control system is the angle of the human joint *q*_*d*_ and the angle sensor placed on the exoskeleton *q*, and the joint torque is as the output of the controller and outputted by the motor driver. It is not necessary and convenient to install an angle sensor on the lower limbs of the human body. Since the angle deviation between the exoskeleton and the human body is usually a constant value, this means we can predict the angle of the human body through the position sensor of the exoskeleton, instead of placing the inertial sensor outside the human body, which is the role of the predict algorithm played in follow-up control strategy.

For the angle data predicted by an algorithm, we used the calculated torque method for systematic control, aiming at making the lower extremity two-link of the exoskeleton follow the changing joint curve predicted by the algorithm. Compared with PD control and PD control with gravity compensation terms, the calculated torque method changes the lower extremity joints of the exoskeleton into a linear time-invariant system that is easier to control due to the introduction of nonlinear compensation. Huo [20] proved the stability of the control method. Based on the inverse dynamics equation, the system can follow the target position well. The control block diagram of this method is shown in Figure 6.

The torque expression calculated by the system control output to the hip and knee joints is as follows:

(20) $$\begin{array}{c} \tau =H\left(q\right)\left(\ddot{q}+K_{d}\dot{e}+K_{p}e\right)+C\left(q,\dot{q}\right)\dot{q}+G\left(q\right). \end{array}$$

In formula (20), the parameters *H*(*q*), $C\left(q,\dot{q}\right)$, and *G*(*q*) are the matrixes of inverse dynamics in the two-link model; *K*_*d*_ and *K*_*p*_ are diagonal matrices, which are proportional and differential terms for the tracking error *e*.

## 3. Results and Discussion

### 3.1. Experimental Results

#### 3.1.1. Prediction Algorithm Experiment Result

Figure 7 represents the sensor data of the motion angle data of the joints in the continuous walking movement. Compared with the sensor data of the wearing exoskeleton, we found that the angle detected from the exoskeleton and the actual motion angle detected from the human body are generally delayed by 200 ms, about 10 sampling cycles. Therefore, in a prediction algorithm, the sensor data at 200 ms after the current sampling point will be predicted based on EXO historical data. The angle sensor data obtained by three participants (65 ± 5 kg, 170 ± 5 cm) continuously walking at a speed of 3.6 km/h on a treadmill was recorded and predicted. None of the participants reported healthy problems in the previous three months.

From the analysis of the accuracy of the prediction angle data shown in Figure 8 and Tables 1 and 2, for both joints, the PSO-Takens has increased the accuracy of the prediction nearly 14.23 ± 0.5% (*n* = 3, two-sided paired *t*-test, *p* = 0 < 0.05), while the smoothing factor is almost unchanged. Due to the fact that the algorithm needs to store historical data, the algorithm will not immediately predict when the algorithm starts to execute. The area where the predicted value is 0 is the dead zone.

Figure 9 and Tables 3 and 4 show the performance of the two prediction algorithms under the standard and fixed frequency of the joint angle (data from [21]). The prediction accuracy in Tables 3 and 4 shows that the accuracy of the prediction is improved (hip joint from 77.85% to 88.19%, knee joint from 87.14% to 95.50%), while the smooth factor remains almost unchanged. Therefore, after the PSO-Takens algorithm is executed, for the movement data of the lower limbs, the prediction algorithm with optimized parameters becomes accurate and stable.

### 3.2. Prediction Algorithm Experiment Result

Since the current pose and the motion-sensing data of the previous period can only reflect the current motion state, to achieve better performance, the exoskeleton system needs to predict the posture data of the following period of time. After processing and analyzing the predicted pose data, the motion intention was judged in advance. By predicting the motion angle of the human body and introducing it into the control of the exoskeleton, the human-machine coordinated motion process of the exoskeleton can be more flexible and smoother.

In order to compare the performance of prediction algorithms and algorithm optimization in simulation, the joint data during motion and the predicted joint data were imported into the two-link model simulation system for a comparative experiment, and the evaluation method of the algorithm mentioned in the second section was used to evaluate the performance of the algorithm. The experimental results are shown in Figure 10.

It can be found that the predicted data lags behind the sensor data of human motion when the system's lower limb joints are controlled to follow the human body at the beginning. Over time, the torque control algorithm with gravity compensation can control the two links to the angle predicted by the two prediction algorithms. When the state or frequency of the motion changes, the prediction error occurs, but the PSO-Takens algorithm shows a better antidisturbance ability, and the maximum error during movement is also better than the original algorithm.

It can be found from Figure 10, in the case of control the movement of the exoskeleton following the lower limbs of the human body without using prediction algorithm, due to the large deviation of the angle, a large interaction force of human-computer interaction force may occur. If the method of prediction is adopted in the control loop of the exoskeleton, the movement of the exoskeleton will be at an angle different from the actual movement of the human body at the initial stage. With the increase of time, the two links of the lower limbs of the exoskeleton gradually follow the movement of the human body and maintain a high consistency with the movement of the human body. It is undeniable that there is still a deviation between the exoskeleton and the human body. According to formula (8), the accuracy of the prediction using the Takens method for hip joint and knee joint is 65.10% and 66.71%, while the PSO-Takens has increased to 82.13% and 83.03%. When the gait becomes stable, the error of Takens algorithms ranges from -0.13 rad to 0.18 rad (hip) and from -0.17 rad to 0.11 rad (knee). While the error of PSO-Takens ranges from -0.04 rad to 0.07 rad (hip) and from -0.05 rad to 0.09 rad (knee).

For standard gait data with a fixed frequency, inappropriate parameters of the Takens algorithm will have obvious errors at the beginning of the prediction, while the PSO-Takens algorithm will not have this problem.  Figure 11 shows that the error of Takens algorithms ranges from -0.14 rad to 0.10 rad (hip) and from -0.12 rad to 0.09 rad (knee), the error of PSO-Takens algorithms ranges from -0.05 rad to 0.06 rad (hip) and from -0.03 rad to 0.04 rad (knee). According to formula (8), the Takens algorithm prediction accuracy rates of the hip and knee joints are calculated as 72.10% and 83.73%, and the PSO-Takens algorithm prediction accuracy rates are 86.07% and 94.01%, which also shows the PSO-Takens algorithm performs better in predicting such data.

## 4. Discussion

In the case of ignoring the elasticity coefficient and inertia coefficient, the human-computer interaction model can be simplified; in this situation, Racine [22] proposed the interaction force can be calculated as follows:

(21) $$\begin{array}{c} F_{e}=K\left(q_{h}-q_{e}\right). \end{array}$$

In formula (24), *F*_*e*_ is the human-machine interaction force and *q*_*h*_, *q*_*e*_ represent the human joint angle and EXO joint angle detected by a sensor, while *K* equals *K*_0_/*L*_0_ (Nm/rad·m), *L*_0_ indicates the distance between the measurement point and the joint rotation center, and *K*_0_ is a constant that varies from the system. Formula (24) means that if there is no angle deviation between the human body and the exoskeleton, it can be considered that the exoskeleton will not hinder the movement of the human body in the walking state of the human body, and the human-machine interaction force will close to 0.

The difficulty of the exoskeleton system controller is how to control the system to move to the target posture of the human body at the next moment. Relying on the installation of an inertial sensor on the exoskeleton has hysteresis and cannot judge the posture of the human body at the subsequent moment. This paper is devoted to the realization of human body motion prediction angle algorithm and introduces it to the control system. The simulation experiment results show that, for the angle prediction of exoskeleton, the PSO-Takens algorithm has the function of improving algorithm parameters. Whether it is linear prediction based on ARMA model LMS, RLS, or DMP [23], the algorithm parameters need to be optimized according to different systems. The PSO-Takens algorithm can deal with periodic during gait walking data, and when the body's movement law changes, such as from walking to jumping or stopping, the accuracy of the prediction algorithm will be reduced, which is the point that the prediction algorithm needs to be improved in the future study.

## 5. Conclusions

In this paper, a human motion capture system is designed to acquire human walking joint data, and a method for optimizing parameters of Takens nonlinear prediction algorithm is proposed. Compared with the original Takens prediction algorithm, the prediction angle obtained by the improved prediction PSO-Takens algorithm is more closely related to the actual motion angle data of the human body, with a smaller error rate and smooth features. When the predicted sensor data from the PSO-Takens algorithm were applied to the joint angle prediction algorithm of the lower extremity exoskeleton, it can improve the accuracy of prediction and enhance the adaptability of the exoskeleton and human body.

## Figures and Tables

**Figure 1:** Motion capture system and exoskeleton structure. (a) Nets of the motion capture system. (b) Motion capture system. (c) Mechanical structure of the exoskeleton.

**Figure 2:** Flow chart of the Takens algorithm.

**Figure 3:** Flow chart of the PSO-Takens algorithm.

**Figure 4:** Lower extremity exoskeleton leg's simplified second link kinetic model.

**Figure 5:** Follow-up control strategy block diagram of the exoskeleton.

**Figure 6:** Control block diagram of calculate torque method.

**Figure 7:** Joint angle deviation between human and exoskeleton.

**Figure 8:** Comparison of Takens and PSO-Takens in prediction of nonstandard gait data. (a) Comparison of hip joint prediction angle. (b) Comparison of knee joint prediction angle.

**Figure 9:** Comparison of Takens and PSO-Takens in prediction of standard gait data. (a) Comparison of hip joint prediction angle. (b) Comparison of knee joint prediction angle.

**Figure 10:** System joint angular output (a). System hip joint angle output (b). System knee joint angle output (c). Hip joint follow control angle error (d). Knee joint follows control angle error.

**Figure 11:** System joint angle output for standard gait data input (a). Hip joint angle output (b). Knee joint angle output (c). Hip joint follow control angle error (d). Knee joint follows control angle error.

**Table 1:** Parameter changes of hip joint prediction algorithm under nonstandard gait data.

#	*T*	*P*	*M*	*L*	PR	SF	Fitness
Takens	10	80	10	300	73.23%	0.2226	38.86
PSO-Takens	10	26	7	644	87.74%	0.2196	46.14

**Table 2:** Parameter changes of knee joint prediction algorithm under nonstandard gait data.

#	*T*	*P*	*M*	*L*	PR	SF	Fitness
Takens	10	80	10	300	71.80%	0.2317	38.05
PSO-Takens	10	48	12	536	85.75%	0.2388	44.97

**Table 3:** Parameter changes of hip joint prediction algorithm under standard gait data.

#	*T*	*P*	*M*	*L*	PR	SF	Fitness
Takens	10	120	10	900	77.52%	0.2133	41.10
PSO-Takens	10	69	3	767	88.19%	0.2091	46.48

**Table 4:** Parameter changes of knee joint prediction algorithm under standard gait data.

#	*T*	*P*	*M*	*L*	PR	SF	Fitness
Takens	10	120	15	900	87.14%	0.2063	45.99
PSO-Takens	10	77	15	1296	95.50%	0.2051	50.18

## Data Availability

The EXO and predicted sensor data based on different algorithms used to support the findings of this study are available from the corresponding author upon request.
